# Observation on the Effect of MRI Image Scanning on Knee Pain in Football Injury

This article has been retracted.

**DOI:** 10.1155/2022/7348978

**Published:** 2022-05-25

**Authors:** Weidong Yu

**Affiliations:** College of Physical Education, Fuyang Normal University, Fuyang, Anhui 236037, China

## Abstract

To study the effect of football injury on knee pain based on MRI image scanning, in this paper, a total of 31 knee injuries of 29 male professional football players from December 2012 to April 2015 were used as the experimental group. The players were 23.6 ± 3.5 years old and received professional football training time 15.3 ± 3.6 years; 31 outpatients of the same age group with acute knee joint acute injury were randomly selected as the control group; both groups were imaged with a 1.5 TMR scanner and knee joint standard array coil imaging, and 2 senior radiation surgeons evaluate knee cartilage, meniscus, ligaments, tendons, bone marrow, infrapatellar fat pad, and joint effusions. Pearson's chi-squared test and nonparametric test for two independent samples were used for statistical testing of the evaluation results. The experimental results showed that there were significant differences in the incidence of articular cartilage, lateral collateral ligament, tendon or ligament injury, multiligament or tendon injury, and bone marrow edema between the two groups (*P* < 0.05). There was no significant difference in the incidence of medial collateral ligament injury, infrapatellar fat pad edema, and joint effusion. MRI shows that knee injuries in male professional football players often involve ligaments or tendons, mostly multiligament or tendon injuries. The lesions of articular cartilage and meniscus are more common and serious, and bone marrow edema is also more common in football injuries. MRI has high diagnostic accuracy for various clinical knee injuries, and it belongs to a noninvasive examination method. It can not only reflect the pathological changes and changes of the knee joints of patients but also provide information for the formulation of clinical programs and the judgment of prognosis, for timely, accurate, and comprehensive imaging reference.

## 1. Introduction

As we all know, in football, players often need to start quickly and in high-speed running, change speed, change direction, stop suddenly, take off, collide, etc. The results of the knee biomechanics study show that the knee strength is the greatest when the knee joint is 30°-50°, so almost all running and jumping movements are also “forced” when the knee is flexed at a 30°-50° angle. In football events where the lower limbs are the main activity, players are required to maintain this position from time to time, the force point is concentrated, and the patellar cartilage surface bears a lot of pressure. At this angle, the contact range of the patella joint is the largest, and the knee is stable at this time. It is mainly maintained by the patella [1]. These anatomical and physiological characteristics have become potential factors for patellar cartilage injury in the semisquatting position. Violent impact and pulling will damage the meniscus and cruciate ligament, causing collateral ligament injury, etc.

As the main weight-bearing joint of the human lower limbs, the knee joint is prone to strain, and with the increase of age, the elderly with chronic diseases have a greater burden on the knee joint and are prone to bone and soft tissue damage (Figure 1) [2]. When people exercise or have a car accident, it is easy to cause injury. The knee joint is a weight-bearing joint in the whole body and is also the most commonly injured joint. With the increase of accidents and injuries, more and more people are injured in the knee joint, but in most people, insufficient attention is paid to knee joint injuries, and the disease is often delayed, so that patients are only admitted to the hospital for treatment when the knee joint function is affected later. At this time, only when the condition of the patient's knee joint is clear can a suitable treatment plan be determined, and the patient's normal knee joint function can be gradually restored. In the diagnosis of knee joint disease, imaging has always been the preferred examination method. Conventional X-ray and CT examinations are more sensitive to bone injuries, but there are many soft tissues around the knee joint, and patients are prone to soft tissue injuries due to accidents. It can not only clarify the patient's bone injury but also better display the soft tissue injury such as the meniscus and the ligaments around the knee joint [3], which is helpful for clinicians to refer to. Among knee joint diseases, MRI gradually shows its incomparable position.

## 2. Literature Review

Malta et al. believe that football is one of the sports with a higher incidence of injury; this is because many technical movements in football, such as strong shooting, falling to the ground, and dribbling, require physical and various muscles. These parts are coordinated and completed together. In addition, the physical confrontation in football is fierce, and the sudden stop and start, jumping, and variable speed running will cause repeated and high-intensity wear and tear to the body, so the sports injury rate in football is relatively high [4]. Endstrasser et al. pointed out in the study that the characteristics of football sports are high intensity, high confrontation, and physical contact. Through the investigation, it is found that the incidence of football injury is from high to low: stomping joint, knee joint, thigh, calf, and medullary joints. Most of the injuries are minor, among which knee stomping joint sprain, thigh muscle strain, and contusion are the most common [5]. Yoon et al. mentioned that the research found that the causes of football players' injuries are mainly caused by insufficient training levels, human factors, and objective factors. Moreover, the incidence of football injuries is on the rise, which should be paid great attention to by athletes and coaches [6]. Anne-Priscille et al. found through a survey of the athletes in the men's football match at the Jilin Provincial University Games that sports injuries in football are mostly concentrated in the lower extremities, of which the stomping joint and knee joint are the parts with a higher incidence of injury, followed by the head, neck, and waist. Fractures mostly occur in the calf; strain in the knee joint and contusion in the lower extremity are relatively high [7]. According to Derouin and others, knee joints are one of the most vulnerable joints in football. Domestic scholars pay more attention to common knee injuries such as medial and lateral collateral ligament injury, meniscus injury, knee cartilage injury, and cruciate ligament injury. The research rate is high [8]. Huang et al. investigated knee injuries in 147 female soccer players from 8 national women's soccer teams in 2006. The results showed that meniscal and knee ligament injuries accounted for the top two cases of total injuries among all female football players participating in the competition [9]. Zhong and Zhu investigated the sports injuries of 8 women's football teams in spring training in 1997 and found that the top three common knee injuries of female football players were knee soft tissue contusion, knee ligament injury, and bone strain [10]. Sun et al. found in their study of football teaching that athletes lack self-protection awareness, lax protection thinking, fail to protect themselves under intense collisions, and also cause knee joint injuries. In football, the force of the knee joint is in the flexion position, and the ligaments of the knee joint are relatively loose in this situation [11]. Pan et al. also studied the injury of the medial and lateral collateral ligaments. The medial and lateral collateral ligaments play a role in stabilizing the knee joint. Compared with the lateral collateral ligaments, the medial collateral ligament has a higher injury rate in football. Direct violence is the main cause of the injury, such as physical confrontation, scramble, and excessive tackle in football games. The athlete's thigh is adducted and internally rotated, and the calf is suddenly abducted and externally rotated. At this time, the medial collateral ligament of the knee joint will be torn or strained. The lateral collateral ligament, on the other hand, is caused by the adduction and internal rotation of the calf and the paradoxical movement of the thigh [12].

## 3. Experimental Analysis

### 3.1. Research Objects

From December 2012 to April 2015, 29 male professional football players (31 knee joints), aged 17 to 29 years, with an average age of 23.6 ± 3.5 years, received professional training for 15.3 ± 3.6 years, all due to knee pain and swelling after training or competition injury, combined with different degrees of dysfunction (experimental group). 31 male patients (31 knee joints, control group) aged 18-30 who underwent MRI examination in the outpatient department of our hospital due to knee joint trauma from May to October 2013 were randomly selected. There was no significant difference in age between the two groups (*F* = 0.01, *P* = 0.971). Those with a history of knee surgery, a diagnosis of knee fracture, or combined systemic diseases (such as rheumatoid arthritis and blood diseases) were not included in this study.

### 3.2. Inspection Method

All subjects were scanned with a 1.5 T dual gradient MR whole-body scanner (Achieva, Philips, The Netherlands), an 8-channel phased coil in the knee joint, and a fast spin echo sequence and a short-time inversion recovery sequence, specifically: sagittal TSE T2WI (TR 3600 ms, TE 100 ms), PD-SPIR (TR 3000 ms, TE 30 ms), coronal TSE T1WI (TR 500 ms, TE17 ms), PD-SPIR (TR 3000 ms, TE30 ms), axial PD-SPIR T2WI (TR3000 ms, TE30ms), slice thickness 5.0 mm, slice spacing 0.5 mm, matrix 512 × 512, and field of view (FOV) 220 mm × 220 mm. The sagittal scan direction is parallel to the running direction of the anterior cruciate ligament, the coronal scan direction is parallel to the femoral condyle, and the axial scan direction is perpendicular to the long axis of the knee joint [13].

### 3.3. Image Analysis

The scanned images were analyzed by 2 experienced radiologists to judge articular cartilage injury, meniscus injury, ligament and tendon injury, bone marrow edema, infrapatellar fat pad edema, joint effusion, etc. For grading, when assessing articular cartilage damage and bone marrow edema, the anatomical sites, namely, lateral tibial plateau, medial tibial plateau, lateral femoral condyle, medial femoral condyle, femoral trochlea, and patella, were analyzed; articular cartilage grading was assessed using the revised Outerbridge grading criteria [14]. The meniscus is divided into medial and lateral meniscus anterior and posterior horns, and the changes are classified into 4 grades using Stoller's criteria. Ligament injuries are classified into three grades: normal ligaments including degenerated ligaments (grade 0), partial ligament tears (grade 1), and completely torn (grade 2). Bone marrow edema is defined as a localized ill-margined signal increase in the bone marrow on lipid-suppressive sequences and a localized ill-defined signal-decreased area on T1WI. Infrapatellar fat pad edema is defined as a hyperintense area with ill-defined margins in the infrapatellar fat pad on T2WI fat-suppressed or proton density-weighted fat-suppressed sequences. The evaluation criteria for joint effusion are that the thickness of the suprapatellar bursa fluid in the anterior-posterior direction on the sagittal plane image is greater than 10 mm, that is, the presence of pathological joint effusion [15].

### 3.4. Statistical Methods

Pearson's chi-squared test was used to compare the knee articular cartilage, meniscus, anterior cruciate ligament, medial collateral ligament, lateral collateral ligament, tendon or ligament injury, multiple ligament or tendon injury, bone marrow edema, and infrapatellar fat pad in the experimental group and the control group. The incidence of edema, joint effusion, and the number of lesions were compared. When *T* < 1, or *n* < 40, or the value obtained after the chi-squared test is close to the test level, the exact probability method is used. The severity of articular cartilage, meniscus, ligament, or tendon lesions was analyzed and compared using nonparametric tests of two independent samples. *P* < 0.05 considered the difference to be statistically significant [16].

## 4. Result Analysis

For the incidence of knee joint injuries, the incidence of articular cartilage, lateral collateral ligament, tendon or ligament injury, multiple ligament or tendon injury, and bone marrow edema in the experimental group was higher than those in the control group. The difference between the two groups was statistically significant, but the meniscus, anterior cruciate ligament injury, medial collateral ligament injury, infrapatellar fat pad edema, and the incidence of joint effusion were not significantly different from the control group (Table 1). For the injury degree, the damaged area (number of lesions) of articular cartilage, meniscus, and tendon in the experimental group was significantly higher than that in the control group. In addition, the degree of articular cartilage and meniscus damage in the experimental group was more serious than that in the control group (Tables 2–4).

From Tables 1–4, it can be seen that knee joint injury seriously affects the training and game quality of football players and even makes some elite athletes end their sports careers prematurely [17–19]. At present, the replantation of articular cartilage is only in the clinical trial stage, and the clinical effect is not exact; it is difficult to recover through conservative treatment after meniscus tear, and it is easy to recur after repair; ligaments and tendons have no regeneration ability and poor healing ability and affect the rupture joint mobility and stability. From Figure 2, timely and accurate diagnosis is helpful for early rehabilitation or surgical treatment, preventing the aggravation of lesions and restoring knee joint function as soon as possible. MRI is used to examine acute and chronic sports-related injuries such as knee cartilage, meniscus, ligaments, and tendons. Check with high consistency.

Football is intense, and the activities and load of the knee joint are large, so it is easy to be damaged. The knee joint is the largest and most complex joint in the human body. The traditional X-ray and CT diagnostic value are limited. Magnetic resonance imaging has high resolution on soft tissue and can image with multiple parameters, multiple orientations, and multiple sequences. The normal meniscus shows a low signal in each sequence. When the meniscus degenerates and tears, it can absorb the synovial fluid in the joint cavity. When the synovial fluid penetrates into the degenerated and torn meniscus, the local proton concentration is increased. T1 and T2 are shortened, so T1 weighting and proton density weighting are more sensitive to meniscus damage [20]. Evaluation of the meniscus is mainly on the sagittal plane on T1 or proton images. Three-dimensional magnetic resonance imaging of the meniscus can clearly show the shape of the meniscus and the location of the injury. The magnetic resonance imaging of meniscus tear shows the following types: (1) oblique meniscus tear: it is the most common type of meniscus tear, and it is generally better in the coronal view than in the sagittal plane; (2) horizontal tear: generally relatively rare, often accompanied by meniscus cysts; (3) barrel-handle tear: more common in young patients with severe trauma, it is a complex tear, and generally, three-dimensional magnetic resonance can show its shape well; (4) radial tear: the direction of tear is perpendicular to the direction of the long axis of the meniscus, and it usually occurs in the lateral meniscus, and it is more common in the inner 1/3 of the meniscus; and (5) longitudinal tear: the direction of the tear is consistent with the direction of the long axis of the meniscus. According to literature reports, with arthroscopy as the standard, the accuracy of MRI diagnosis of meniscus is 90% to 100%.

As a noninvasive examination, MRI has high tissue resolution and can correspond to pathology and arthroscopic grading. The meniscus injury is divided into three grades according to its shape and degree: the first grade is an amorphous or spherical high signal shadow; the second grade is a linear high signal shadow, neither of which extends to the articular surface; and the third grade is linear or diffuse hyperintensity extending into the articular surface representing an arthroscopic tear [21]. In order to reduce the false-positive rate, a high-intensity shadow extending to the meniscus surface must be seen on both the coronal and sagittal planes to diagnose a tear. Among ligament injuries, the anterior cruciate ligament is more common than the posterior cruciate ligament, and the medial collateral ligament is more common than the lateral collateral ligament. Common MRI findings of ligament tears include the following.

### 4.1. Direct Signs

(1) No normal ligaments can be seen on the coronal and sagittal planes, (2) the ligaments are interrupted and discontinuous, (3) the ligaments are thickened with irregular or wavy edges, and (4) there is a localized or diffuse high signal in the ligaments.

### 4.2. Indirect Signs

The indirect signs are (1) avulsion fracture at the ligament attachment, (2) local cartilage defect or with meniscus tear, and (3) bone contusion and bone marrow edema.

In addition, it may be accompanied by bursae effusion, subcutaneous tissue, fascial edema, and disappearance of nearby fat shadows. The presence or absence of edema in the ligament and its adjacent soft tissues is the main basis for identifying acute and chronic injuries. In judging the bone condition after trauma, plain X-ray still has an irreplaceable role, but MRI has certain advantages in showing the hidden lesions of the knee bone structure because it can select a variety of sequences [22]. It can be used as an important supplement to determine the bone condition of X-ray plain film. The MRI of occult bone lesions of the knee joint can be divided into five types: type I: long T1 and long T2 signal areas with blurred long T1 and long T2 signals in the bone or metaphysis, with unclear boundary and irregular shape, which reflect the bone marrow edema of pure bone contusion [23, 24]. Type II: line-like structures with mixed signals of high and low signals are seen in type I lesions and extend to the cortex, and the corresponding cortical lines are slightly staggered, reflecting an occult fracture. Type III: there is a patchy, fuzzy high signal area on T1WI and T2WI immediately under the articular cartilage, and a line-like structure extending to the cartilage can be seen, indicating an osteochondral joint injury. Type IV: T1WI and T2WI are hypointense lesions immediately under the articular cartilage, with clear borders, and the thickness, shape, and signal of the upper cartilage may have different degrees of change, suggesting subosseous bone sclerosis. Type V: the subchondral bone structure of the articular cartilage shows a low signal on T1WI, T2WI shows a central high-peripheral low signal shadow, with clear boundary and abnormal changes in the cartilage on the lesion, because the structure is continuous with the diseased cartilage, so it may be due to a cartilage break invasion of synovial fluid and synovium. Types I to III are more common in acute injuries, and types IV to V are more common in chronic injuries. Among the hidden intraosseous lesions, the tibia is the most common site and is often associated with articular ligament injury, especially the anterior cruciate ligament. MRI can clearly show the effusion of the knee joint cavity and can distinguish the composition of the fluid according to the different signals [25]. In this article, there are 3 cases of lipemia in the joint cavity, which is caused by the simultaneous entry of adipose tissue and blood from the bone marrow cavity or the torn periosteum into the joint cavity after trauma, and the fat floats on the synovial fluid, and the blood submerged under the synovial fluid; MRI showed three layers of joint effusion with different signals.

## 5. Conclusion

The injury of the meniscus and articular cartilage of the knee joint of football players is more serious and involves multiple structures of the knee joint, which is consistent with the research of other scholars. Cartilage signal changes were seen in 11 joints in the athletes in this group, of which 4 had full-thickness loss of cartilage and exposed subchondral bone. In addition to articular cartilage damage, these 4 were combined with severe damage to other structures, while none of the control group had joints. For full-thickness exfoliation of cartilage, articular cartilage damage is considered to be the core pathological change of osteoarthritis, which is more common in middle-aged and elderly people, but repeated and intense trauma can also cause articular cartilage rupture and peeling in adolescents. Among the 31 knee joints in the experimental group, there were 11 knee joints with third-degree injury of the meniscus, 12 with second-degree injury, and 9 with first-degree injury. Since the course of the knee joint is mostly acute, it is recommended that for acute knee joint injury, early diagnosis and early treatment must be performed, so that the injury can heal as soon as possible and to prevent the acute injury from turning into a chronic injury.

To sum up, MRI imaging examination for knee joint injury can reduce the radiation to the patient and can clearly identify the pathological changes in the knee joint of the patient. The evaluation of late prognosis provides imaging reference, which is worthy of promotion and application in clinical practice.

## Figures and Tables

**Figure 1:** Knee sports injury.

**Figure 2:** The relative *P* value of the knee joint of the experimental group and the control group (cases).

**Table 1:** Comparison of the incidence of knee joint injury between the experimental group and the control group (case (%)).

Group	Meniscus	Cartilage	Anterior cruciate ligament	Medial collateral ligament	Lateral collateral ligament	Hamstrings
Test group	16	11	12	17	14	6
Control group	11	4	14	13	5	1
*P* value	0.200	0.038	0.607	0.309	0.013	∗

**Table 2:** Statistical table of the distribution of knee cartilage injury in the experimental group and the control group (cases (%)).

Group	Lateral tibial plateau	Medial tibial plateau	Lateral malleolus of femur	Medial malleolus of femur	Femoral trochlea
Test group	6	6	4	4	4
Control group	2	2	0	2	0
*P* value	∗	∗	∗	∗	∗

**Table 3:** Statistical table of the distribution of knee meniscus injury in the experimental group and the control group (cases (%)).

Group	Medial meniscus		Lateral meniscus		Total
	Front corner	Rear corner	Front corner	Rear corner	
Test group	4	8	18	4	34
Control group	1	2	7	5	15
*P* value	∗	0.038	0.004	0.718	0.002

**Table 4:** Statistical table of grading of knee articular cartilage, meniscus, and tendon lesions in experimental group and control group (cases).

		Level 0	Level 1	Level 2	Level 3	Level 4	*P* value
Articular cartilage	Test group	158	12	9	3	4	0
	Control group	179	2	3	2	0	
Meniscus	Test group	90	11	12	11	—	0
	Control group	109	3	3	9	—	
Tendon or ligament	Test group	—	52	13	—	—	—
	Control group	—	35	9	—	—	

## Data Availability

The data used to support the findings of this study are available from the corresponding author upon request.
